RETRACTED

# Enhanced Immune Response and Protective Effects of Nano-chitosan-based DNA Vaccine Encoding T Cell Epitopes of Esat-6 and FL against *Mycobacterium Tuberculosis* Infection

**DOI:** 10.1371/journal.pone.0061135

**Published:** 2013-04-23

**Authors:** Ganzhu Feng, Qingtao Jiang, Mei Xia, Yanlai Lu, Wen Qiu, Dan Zhao, Liwei Lu, Guangyong Peng, Yingwei Wang

**Affiliations:** 1 Department of Microbiology and Immunology, Nanjing Medical University, Nanjing, China; 2 Department of Pathology, Hong Kong University, Hong Kong, China; 3 Division of Infectious Diseases, Allergy and Immunology, Department of Internal Medicine, Saint Louis University School of Medicine, St. Louis, Missouri, United States of America; Glaxo Smith Kline, Denmark

## Abstract

Development of a novel and effective vaccine against *Mycobacterium tuberculosis* (*M.tb*) is a challenging for preventing TB infection. In this study, a novel nanoparticle-based recombinant DNA vaccine was developed, which contains Esat-6 three T cell epitopes (Esat-6/3e) and fms-like tyrosine kinase 3 ligand (FL) genes (termed Esat-6/3e-FL), and was enveloped with chitosan (CS) nanoparticles (nano-chitosan). The immunologic and protective efficacy of the nano-chitosan-based DNA vaccine (termed nano-Esat-6/3e-FL) was assessed in C57BL/6 mice after intramuscular prime vaccination with the plasmids DNA and nasal boost with the Esat-6/3e peptides. The results showed that the immunized mice remarkably elicited enhanced T cell responses and protection against *M.tb H37Rv* challenge. These findings indicate that the nano-chitosan can significantly elevate the immunologic and protective effects of the DNA vaccine, and the nano-Esat-6/3e-FL is a useful vaccine for preventing *M.tb* infection in mice.

## Introduction

Tuberculosis (TB) infected by *Mycobacterium tuberculosis (M.tb)* has plagued humankind worldwide for many years [1]. Although bacillus Calmette-Guerin (BCG) is an effective vaccine for childhood TB, it produces incomplete and variable protection in adult TB [2]. Furthermore, BCG is also an attenuated vaccine that cannot be safely given to the persons infected with human immunodeficiency virus (HIV). Thus, a new and efficient vaccine against TB is urgently required.

Control of *M.tb* infection greatly depends on T cell-mediated immune responses [3]. The 6 kDa early secretory antigenic target (Esat-6), which presents in virulent mycobacterial strains and absents in BCG [4], is critical for *M.tb* immunogenicity and virulence. Because Esat-6 protein can be recognized by T cells and B cells [5], and it has attracted intense interests in vaccine development. Given that *M.tb* Esat-6 gene is located in virulent *M.tb* [6], avoiding Esat-6 adverse reaction in the vaccine studies is also indeed important.

RETRACTED

It has been reported that the DNA vaccines based on T cell epitopes of *M.tb* antigens can induce efficient immune responses, and decrease side effects and increase safety and stability of vaccines [7], [8]. However, DNA poor delivery to antigen presenting cells (APCs) and the rapid inactivation mediated by DNase results in low immunogenicity of DNA vaccines [9]. Thus, elevating DNA vaccine delivery efficiency of DNA vaccine and protecting DNA from degradation are important for enhance DNA vaccine potency.

Several documents have reported that fms-like tyrosine kinase 3 ligand (FL) plays an important role in proliferation and differentiation of myeloid and lymphoid progenitor cells as well as dendritic cells (DCs) [10]. Moreover, FL has a strong adjuvant effects that augment DC recruitment and expansion, as well as increase antigen uptake and cross presentation [11], [12].

Chitosan (CS) is a non-toxic biodegradable and biocompatible polycationic polymer, which can not only bind DNA and protect it from nuclease degradation [13], [14], [15], [16], but also exhibit potential adjuvant properties, such as promoting endocytotic uptake and elevating immune responses. Additionally, chitosan nanoparticles (nano-chitosan) possess lower cytotoxicity and more stability [17], [18], [19], [20], [21].

In order to evaluate the immunologic and protective efficacy of CS nanoparticle-based DNA vaccine expressing T cell epitopes of Esat-6 and FL against *M.tb* infection, in the present study, the three T cell epitopes of Esat-6 (Esat-6/3e) were predicted and selected based on the pitope prediction software analyses. Then, a recombinant plasmid DNA vaccine that contains the genes of Esat-6 three T cell epitopes (Esat-6/3e) was constructed and identified. Subsequently, the recombinants were enveloped with nano-chitosan, and the nano-chitosan-based recombinants were identified, and validated the expression in rat glomerular mesangial cells (GMCs). More importantly, the immunologic and protective effects against *M.tb* infection mediated by the nano-chitosan-based DNA vaccines were evaluated *in vivo* in mouse models.

## Results

### Prediction of T cell epitopes and identification of recombinant Esat-6/3e-FL plasmid

Based on MHC-binding scores of the MHCpre software analyses (http://www.syfpeithi.com/scripts/MHCSr.dll/home.htm; http://tools.immuneepitope.org) and literatures [22], the three T cell epitopes of Esat-6 were selected for the DNA vaccine development as follow: Esat-6_4–18_ (QQWNFAGIEAAASAI), Esat-6_22–36_ (VTSIHSLLDEGKQSL) and Esat-6_56–70_ (QKWDATATELNNALQ). To protect the epitopes against amalgamation and enhance efficacy of intracellular protease incising [23], the Ala-Ala-Tyr (AAY) linker and a his tag were inserted into pIRES (vector) and pIRES-FL plasmids, named pIRES-Esat-6/3e (Esat-6/3e) and pIRES-Esat-6/3e-FL (Esat-6/3e-FL), respectively (Figure 1A.). To verify whether the recombinant plasmids can express the corresponding protein, the plasmids were transfected into rat GMCs for 60 h, and the expression of his tag and FL protein was determined by Western blot (Figure 1B).

RETRACTED

**Figure 1:** Construction and identification of pIRES-Esat-6/3e-FL (namely Esat-6/3e-FL). **A.** Schematic representation of Esat-6/3e-FL. **B.** The expression of his tag and FL proteins from Esat-6/3e or Esat-6/3e-FL plasmids was determined using Western blot after transfection of the plasmids into rat GMCs for 60 h (1: pIRES-Esat-6/3e. 2: pIRES-Esat-6/3e-FL. 3: pIRES-FL. 4: pIRES). **C.** The irregular solid spheres of nano-chitosan and nano-Esat-6/3e-FL plasmids under EM. **D.** The expression of his or FL proteins from the Esat-6/3e-FL plasmids enclosed with chitosan nanoparticle (nano-Esat-6/3e-FL) was confirmed using Western blot with anti-his or anti-FL antibody at 60 h after transfection into rat GMCs (1: MEM. 2: nano-pIRES. 3: nano-Esat-6/3e-FL).

### Diameter, zeta potential and shape of nano-chitosan and nano-Esat-6/3e-FL plasmids

The diameter and dispersing degree of nano-chitosan particles were 311.2±34 nm and 0.35 respectively. Their zeta potential was 30.6 mV. After the recombinant Esat-6/3e-FL plasmids were coated with nano-chitosan (nano-Esat-6/3e-FL), the diameter and zeta potential of the nano-plasmids were 314.8±38 nm and 33.6 mVseparately, and their dispersing degree was 0.39 (Figure S1A, and S1B). Moreover, the particles of nano-chitosan and nano-Esat-6/3e-FL displayed an irregular solid sphere, and their diameters were from 280 to 330 nm (Figure 1C).

### Stability, transfection efficacy and expression of nano-Esat-6/3e-FL plasmid

The nano-Esat-6/3e-FL plasmids were first digested by different concentrations of DNase I. When agarose gel electrophoresis was performed, the Esat-6/3e-FL plasmid DNAs departed from the sample well, but the corresponding nano-plasmids stayed in the well (Figure S2A). The different volume ratio of nano-chitosan and Esat-6/3e-FL mixture was digested by the same dose of DNase I. The results manifested that Esat-6/3e-FL plasmids were well digested when the ratio was at 1∶4 (Figure S2B). In addition, the transfection efficiency and cytopathic effect of pGCsi-GFP enveloped by nano-chitosan (nano-chitosan-GFP) or liposome-2000 were observed in rat GMCs. The results confirmed that the CPE of GMCs transfected with nano-chitosan-GFP at 48 h or 72 h was markedly lower than that of GMCs transfected with pGCsi-GFP coaded by liposomes-2000 (Figure S3). Moreover, the nano-Esat-6/3e-FL plasmids could also express the corresponding proteins (Figure 1D).

RETRACTED

### Production of cytokines and expression of T-bet, Gata-3 from the splenocytes of the nano-Esat-6/3e-FL-immunized mice

In order to evaluate T cell immune responses elicited by the nano-Esat-6/3e-FL vaccination, splenocytes from the immunized mice were collected and cultured. The amounts of IFN-γ, IL-12, IL-4 and IL-10 in the supernatant were detected by ELISA. The levels of IFN-γ and IL-12 in the mice vaccinated with nano-Esat-6/3e-FL or nano-Esat-6-FL were obviously higher than those with other plasmids, which even exceed the levels in BCG treatment group.Furthermore, mice immunized with nano-Esat-6/3e-FL elicited much higher levels of IFN-γ and IL-12 than those immunized with Esat-6/3e-FL. However, the levels of IL-4 and IL-10 from the mice vaccinated with BCG were the highest among all the vaccinated mice (Figure 2A). In addition, the expression levels of T-bet mRNA and protein in nano-Esat-6/3e-FLimmunized mice were obviously higher than those in the other groups treated with other plasmids or BCG (Figure 2B). However, Gata-3 mRNA and protein expressions did not show obvious changes among all the groups. These results suggested that the mice immunized with nano-Esat-6/3e-FL and nano-Esat-6-FL could induce a stronger Th1-polarized response.

**Figure 2:** Splenocytes of the mice immunized with different plasmids were cultured and stimulated with Esat-6/3e (10 µg/ml) for 72 h, and the production of IFN-γ, IL-12, IL-4 and IL-10 in the splenocyte supernatants and expression of T-bet and Gata-3 in the splenocytes were measured by ELISA and Western blot, respectively. **A.** The levels of Th1 type cytokines (IFN-γ and IL-12) and Th2 type cytokines (IL-4 and IL-10). **B.** The expression levels of T-bet or Gata-3 mRNA and protein. The representative graph and histograms in the immunized mice were showed. The experiments were performed in three times. All data are from one representative of three experiments, and presented as the mean value ± SD (n = 6). The statistics were performed with one-way ANOVA. *NS: P*>0.05; *P<0.05 and ***P<0.001 versus the mice with nano-chitosan, nano-pIRES and nano-FL immunization respectively. The other significant differences among the mice vaccinated with nano-Esat-6/3e-FL, nano-Esat-6/3e, Esat-6/3e-FL, nano-Esat-6, nano-Esat-6-FL and BCG were displayed on the figure directly.

### Proliferation of spleen cells and numbers of IFN-γ^+^ T cells from the nano-Esat-6/3e-FL immunized mice

To verify the efficacy of immunologic reaction induced by nano-Esat-6/3e-FL vaccination, proliferation of spleen cells from the immunized mice was detected. As shown in Figure 3A, the SI increased more conspicuously in the mice with nano-Esat-6/3e-FL vaccination than that in other groups. The SIs of the mice treated with nano-Esat-6-FL and BCG were also significantly elevated, but no marked difference, compared with the nano-Esat-6/3e-FL immunization group.

RETRACTED

**Figure 3:** The proliferation of the splenocytes and number of IFN-γ^+^ T cells of the mice immunized by nano-Esat-6/3e-FL. **A.** Splenocytes were cultured and stimulated with the Esat-6/3e (10 µg/ml) for 72 h. The stimulation index (SI) of splenocytes in the mice treated with different vaccines was calculated to determine the proliferation activity. **B.** The numbers of IFN-γ^+^ T cells from the splenocytes were quantified by ELISPOT assays. Data are one representative of three experiments and presented as mean value ± SD (n = 6). The statistics were performed with one-way ANOVA. *NS: P*>0.05; ***P<0.001 versus the mice treated with nano-chitosan, nano-pIRES and nano-FL plasmids. The differences among other treatments were shown directly on the figure.

To further determine whether the nano-Esat-6/3e-FL can trigger high T cell responses, IFN-γ –producing T cells of immunized mice were evaluated using ELISPOT assays. IFN-γ^+^ T cell numbers (spot forming cell, SFC) in the mice with nano-Esat-6/3e-FL vaccination were much higher than those in the mice immunized with Esat-6/3e-FL. Although IFN-γ^+^ T cell numbers in the mice immunized with nano-Esat-6-FL were the highest, there was no significant difference in comparison to the mice immunized with nano-Esat-6/3e-FL vaccine (Figure 3B).

### CTL activity of mice triggered by nano-Esat-6/3e-FL immunization

To assess the cytolytic capability of CTLs induced by nano-Esat-6/3e-FL vaccination, an *in vivo* cytotoxicity assay was performed. As shown in Figure 4, a significantly increased lyses were founded in the mice immunized with nano-Esat-6/3e, Esat-6/3e-FL, nano-Esat-6 or nano-Esat-6-FL separately (Figure 4). In addition, much higher cytolytic activity was observed in the mice immunized with nano-Esat-6/3e-FL or nano-Esat-6-FL, though there was no significant difference between these different groups, which also overtopped markedly BCG vaccination.

**Figure 4:** The CTL activity of the mice elicited by nano-Esat-6/3e-FL or other plasmids. Splenocytes from naive mice pulsed with (CFSEhigh) or without (CFSElow) peptides were transferred into the immunized mice. The representative histograms (**A**) and percentages (**B**) of specific lysis in the immunized mice were compared. Data are one representative results from three performed experiments, and presented as the mean ± SD (*n* = 6). *NS: P*>0.05; *P<0.05; ***P<0.001 versus the mice treated with nano-chitosan, nano-pIRES or nano-FL plasmids; the other differences among nano-Esat-6/3e-FL, nano-Esat-6/3e, Esat-6/3e-FL, nano-Esat-6, nano-Esat-6-FL and BCG treatments were showed on the figure directly.

RETRACTED

### Protective effects against *M.tb* H37Rv challenge from the mice immunized with nano-Esat-6/3e-FL

To determine the protective potential of nano-Esat-6/3e-FL vaccination, one week after the last boost with Esat-6/3e peptides, the vaccinated mice were intratracheally challenged with 1×10^6^ bacilli *M.tb* H37Rv. The bacterial burdens in the lungs and spleens, including pulmonary injury were observed at 4 weeks post challenge. As shown in Figure 5, the reduction of *M.tb* colonies was significantly observed both in the lungs (Figure 5A) and spleens (Figure 5B) in the mice with nano-Esat-6/3e-FL immunization, and the value of log_10_ CFU was 0.403±0.023 and 0.324±0.062, respectively, although the log_10_ CFU value in the mice vaccinated with nano-Esat-6/3e-FL plasmids was similar to that of the mice treated with nano-Esat-6-FL plasmids. Meanwhile, the burden of log_10_ CFU in the lungs from these two groups was sharply decreased compared with that from BCG vaccination. These findings indicated that immune responses of the mice induced by nano-Esat-6/3e-FL (including nano-Esat-6-FL) plasmid DNA vaccine could indeed lead to an enhanced defense.

**Figure 5:** The protection efficacy against *M.tb* infection of the mice immunized with different vaccines. Mice vaccinated with different plasmids and boosted with Esat-6/3e peptides for two times were infected with 1×10^6^ bacilli of *M.tb* H37Rv for 4 weeks. Bacterial loads in the lungs (**A**) and spleens (**B**) of these mice were examined and the sections of the lung tissues from these mice were performed HE staining. Representative histologic changes (100×) depicted the lung tissue of the infected mice (**C**).

On the other hand, the lung tissues of the mice vaccinated with nano-chitosan, nano-pIRES and nano-FL showed widespread and severe interstitial pneumonia including larger diffuse granuloma and infiltration of inflammatory cells after *M.tb* H37Rv infection, while the mice immunized with nano-Esat-6/3e-FL (including nano-Esat-6-FL or BCG) displayed moderate damage with relatively fewer cell infiltration, smaller granulomas and better lung structure (Figure 5C).

Additionally, to determine whether the mice immunized with nano-Esat-6/3e-FL affect the influx of T cells and macrophages, the lung sections were stained with anti-CD3 or anti-F4/80 antibody. The results displayed that the numbers of CD3 (Figure S4A) and F4/80 (Figure S4B) positive cells in the mice immunized with nano-Esat-6/3e-FL were much more than the mice from other treatment groups. Furthermore, the mice treated with nano-Esat-6/3e-FL possessed more intact alveolar tissue, implicating the inflammatory changes mediated by *M.tb* were attenuated (Figure S4C). These results suggest that the nano-chitosan-based DNA vaccine could induce a strong and effective protection against *M.tb* challenge in the immunized mice.

RETRACTED

## Discussion

Previous studies have reported that one of major contributors to the virulence and intercellular spread of *M.tb* is Esat-6 secretion system 1 (ESX-1) that is lost in BCG [24], [25], [26], [27], [28]. In addition, Esat-6 also contains a large number of antigen epitopes recognized by T and B cells. Immunization with Esat-6 in mice not only induces highlevels of IFN-γ and low bacterial loads after *M.tb* challenge [29], [30], [31], [32], [33], [34]. Since epitope vaccines can overcome safety problem and induce potent immune responses [35]–[37], in our previous [38] and present studies, three T cell epitopes of Esat-6 (Esat-6_4–18_, Esat-6_22–36_ and Esat-6_56–70_), which contain Th1 and/or CTL epitopes [39]–[42], were selected according to higher scores via prediction software analyses.

In view of relatively low immunogenicity of DNA vaccine [13], the strategy of increasing delivery efficiency and protecting DNA from degradation may elevate the protective effects. FL is used as an effective adjuvant due to its enhancing antigen presentation [21]. Furthermore, in our previous experiments [38], co-delivery of FL for ESAT-6 epitopes DNA vaccines was confirmed to remarkably increase the efficacy of immunity and protection in mice.

It has been known that chitosan (CS) can effectively bind to DNA and protect it from nuclease degradation, and DNA packaged with nano-chitosan can improve cell uptake and vaccine delivery [13], [14], [15], [16], [41], [43], [44], [45], [46], [47]. In the present study, the recombinant candidate plasmid that contained 3 T cell epitopes and FL (pIRES-Esat-6/3e-FL), as well as the recombinant control plasmids i.e. pIRES-Esat-6/3e, pIRES-Esat-6 (containing full length of ESAT-6) and pIRES-FL (only containing FL) were first constructed and then enclosed with nano-chitosan. Our results showed that the nano-chitosan-based plasmids could transfect into GMCs and the corresponding protein was effectively expressed. Although the mice immunized with the control plasmids and BCG obviously elevated T cell responses and CTL activities, much more responses and effects were observed in the mice vaccinated with nano-Esat-6/3e-FL. Moreover, those immunized mice displayed remarkably protective efficacy, including the inhibition of *M.tb* growth and lung damage, but the better effects were seen in the mice immunized with nano-Esat-6/3e-FL and nano-Esat-6-FL, implicating that FL and nano-chitosan generated a markedly synergistic role as immune adjuvant for the DNA vaccine. Since lower cytotoxicity of nano-Esat-6/3e plasmid was demonstrated in rat GMCs, thus we think that the nano-Esat-6/3e plasmid DNA might be a better vaccine.

RETRACTED

On the other hand, the mice vaccinated with BCG could not only induce high levels of IFN-γ and IL-12, increased T-bet expression and IFN-γ^+^ T cells and augmented CTL activity, but also provide strong protection. However, the immune response efficiency of the mice with BCG immunization were relatively lower than that of the mice with nano-Esat-6/3e-FL (including nano-Esat-6-FL) vaccination, indicating that the nano-Esat-6/3e-FL DNA vaccine can mediate more powerful T cell responses and may be superior to BCG. Furthermore, since the pathological changes of mice vaccinated with nano-Esat-6/3e-FL were markedly lower than those of the mice treated with nano-whole Esat-6 and FL (nano-Esat-6-FL), we consider that the plasmid DNA vaccine encapsulated with nano-chitosan (nano-Esat-6/3e-FL) is relatively better than nano-Esat-6-FL plasmid DNA.

Reportedly, Bennekov' study [48] showed that the adenoviral construct induced a strong CD8 response predominantly targeted to the epitope Esat-6_15–29_, but there was no significant protection against *M.tb* infection. Thus, in our current experiment, we selected the three epitopes (Esat-6_4–18_, Esat-6_22–36_ and Esat-6_56–70_) that based on the computer prediction. Our results demonstrated that the mice immunized with nano-Esat-6/3e-FL plasmid DNA vaccine not only elicited enhanced T cell responses, but also remarkably elevated the protection against *M.tb* challenge.

Additionally, it is worth mentioning that *in vitre* experiment, the splenocytes had also been stimulated with PPD, but the data (not shown) were similar to data of the splenocytes with Esat-6/3e peptides. Ergo, to demonstrate the increased antigen-specific immune responses, we used the data from the epitope peptides stimulation in the paper. In terms of such amount of IL-10 and IL-4 (look higher) in nano-chitosan, nano-pIRES and nano-FL (see Fig. 2), here we explain that IL-10 and IL-4 have a basic level in mice, while the relatively lower levels of IL-10 and IL-4 in the mice treated with the plasmid vaccines might be related with elevated Th1 and decreased Th2 responses. However, the mechanisms need to be explored in the future.

RETRACTED

In summary, our data demonstrated that the selected three T cell epitopes of Esat-6 were dominant epitopes for Th1 cells and CTLs which can significantly increase Th1 polarization reactions and CTL activity. Moreover, FL is a critical immunostimulatory adjuvant that promoted more strong immune responses and protection against *M.tb* induced by DNA vaccines. More importantly, nano-chitosan could also significantly enhance the vaccination effects of Esat-6/3e-FL DNA vaccine, such as strong Th1 and CTL immune responses and inhibition of *M.tb* growth. Collectively, our findings indicate that the nano-chitosan-based DNA vaccine (nano-Esat-6/3e-FL) is a novel and useful tool for preventing *M.tb* infection.

## Materials and Methods

### Animals

Eight-week-old female C57BL/6 mice (H-2^b^) were purchased from the central animal laboratory of Yangzhou University (China), and maintained under specific pathogen-free conditions (eight in each group). All the experiments were conducted according to the Institutional Ethical Guidelines for Animal Experiments of Nanjing Medical University (permit number: 2010257).

### T cell epitope prediction, plasmid construction and identification

The plasmids of pIRES-Esat-6-FL (containing full length of Esat-6 and FL) and pIRES-Esat-6 (only containing full length of Esat-6) as well as pIRES-FL (only containing full length of FL) have been previously described [7] and kept in our lab. The primary structure of Esat-6 antigen was analyzed by epitope prediction software online (http://www.syfpeithi.com/scripts/MHCSr.dll/home.htm; http://tools.immuneepitope.org). Three T cell epitopes, namely Esat-6_4–18_ (QQWNFAGIEAAASAI), Esat-6_22–36_ (VTSIHSLLDEGKQSL) and Esat-6_56–70_ (QKWDATATELNNALQ) were sorted based on their scores [38]. A his tag, the three peptides and Ala-Ala-Tyr (AAY) linker were synthesized and inserted into pIRES or pIRES-FL plasmids, which were termed pIRES-Esat-6/3e (Esat-6/3e) and pIRES-Esat-6/3e-FL (Esat-6/3e-FL). Thereafter, these plasmids were prepared and purified with endoFree plasmid maxi kit (Qiagen, Germany) and transfected into rat GMCs. Subsequently, the expression of his and FL protein of these plasmids was detected using Western blot [38].

### Chitosan nanoparticle, nano-plasmid DNA preparation and identification

Chitosan (CS) was purchased from Treechem. Ltd (Shanghai, China), and dissolved in 1% acetic acid and mixed with 0.1% pentasodium triphosphate (TPP), then the formation of chitosan-TPP nanoparticles started spontaneously via the TPP initiated ionic crosslink and coacervation [21]. To get mixture of nano-chitosan and plasmid DNA, both prepared nano-chitosan and plasmid DNA suspension heated and mixed in different volume. Thereafter, the particle size, zeta potential and polydispersity of nano-chitosan and nano-Esat-6/3e-FL plasmids were measured by a Malvern Zetasizer 3000-HS at 633 nm. The morphological shape of the nanoparticles was observed by electron microscopy (EM).

RETRACTED

The suspensions of nano-chitosan and nano-plasmid DNA were separated by ultra centrifugation. The amount of free-DNA in the supernatant was detected at 595 nm, and the DNA encapsulation efficiency (EE) was calculated using Eq: EE = (total amount DNA–free amount DNA in supernatant)/total amount DNA×100%. Meantime, different gradient amount of DNase I (0.02U, 0.04U and 0.1U) was added into the naked plasmid DNA and nano-plasmid DNA with the same quantity for 15 min. The mixture was electrophoresed with 2% agar. Furthermore, these plasmids were transfected into glomerular mesangial cells (GMCs) separately and cultured for 60 h. Thereafter, the lysate of GMCs was electrophoresed on SDS-PAGE gels, and stained with anti-his or anti-FL mAb (Santa Cruz, USA).

### Esat-6 peptide, BCG and *M.tb* H37Rv preparation

The Esat-6 peptides (Esat-6/3e) comprising the 3 T cell epitopes were synthesized by Sangon Biotech Co. Ltd (Shanghai, China), and confirmed to be of >90% purity by high-performance liquid chromatography and mass spectrometry profiles. BCG (Denmark strain 1331) was provided by Center for Disease Control of Jiangsu Province in China. A virulent *M.tb* H37Rv strain (ATCC 27294) supplied by National Institute for the Control of Pharmaceutical and Biological Products (Beijing, China) was grown in 7H9 liquid medium supplemented with albumin-dextrose-catalase enrichment.

### Vaccine immunization and *M.tb* H37Rv challenge

All female C57BL/6 mice housed in specific pathogen free conditions, and were randomly assigned to 9 groups (eight in each group) as shown in Table 1. To compare the different effects on T cell immune response in the mice immunized various relative materials, the mice of candidate group were treated with nano-Esat-6/3e-FL plasmid DNA. And the mice of control groups treated with nano-Esat-6/3e, nano-Esat-6-FL, nano-Esat-6, nano-FL, nano-chitosan, nano-pIRES, Esat-6/3e-FL and BCG, respectively. In nano-plasmids treatment, the mice were injected intramuscularly three times at 3-week intervals in both quadriceps muscles with 100 µl nano-chitosan or 100 µl different nano-plasmids (containing 100 µg DNA, separately). In Esat-6/3e-FL treatment, the mice were vaccinated with 100 µl Esat-6/3e-FL plasmids (containing 100 µg DNA) without nano-chitosan envelopment. In BCG treatment, the mice were injected subcutaneously with 10^6^ BCG only once at equal pace. Three weeks after two immunizations, the mice were dripped via airway with 25 µg Esat-6/3e peptides two times at 1-week interval. In order to induce higher immune responses, the animals were boosted [49], and 2 weeks after the last peptides boost, parts of mice were euthanized for testing immune response, and the remaining mice were challenged intratracheally with 100 µl (10^6^ bacilli) of *M.tb* H37Rv per animal. Four weeks post *M.tb* challenge, these mice were sacrificed for bacterial burdens and histological assessment [48]. The whole schedule of vaccination in mice was displayed in Figure 6.

RETRACTED

**Figure 6:** Sketch drawing of immunization procedure and challenge by *M.tb* H37Rv. **A.** C57BL/6 mice were injected intramuscularly three times at 3-week intervals in both quadriceps muscles with different nano-plasmids, nano-chitosan, Esat-6/3e-FL or BCG. Those mice were then boosted with Esat-6/3e peptides through intranasal administration once a week for 2 weeks, then sacrificed at 1 week after the last peptide boost. **B.** Mice vaccinated with different nano-plasmids for 3 times and boosted with Esat-6/3e peptides for 2 times as above mentioned time schedules were infected with *M.tb* H37Rv the airway at 1 week after the last peptide boost, and then sacrificed at 4 weeks post *M.tb* H37Rv challenge.

**Table 1:** The groups of mice given with different treatments.

	Esat-6/3e	Esat-6	FL	pIRES	nano-chitosan	BCG
**Candidate group**						
nano-Esat-6/3e-FL	+	−	+	+	+	−
**Control group**						
nano-Esat-6/3e	+	−	−	+	+	−
nano-Esat-6-FL	−	+	+	+	+	−
nano-Esat-6	−	+	−	+	+	−
nano-FL	−	−	+	+	+	−
nano-chitosan	−	−	−	−	+	−
nano-pIRES	−	−	−	+	+	−
Esat-6/3e-FL	+	−	+	+	−	−
BCG	−	−	−	−	−	+

### Cytokines, T-bet and Gata-3 detection

The spleen cells from immunized mice were cultured on plates at 2.5×10^5^ per well, and then incubated with the Esat-6/3e peptides (10 µg/ml) for 72 h. The levels of IFN-γ, IL-12, IL-4 and IL-10 in the supernatants were determined by ELISA (Biolegend, USA). In addition, total RNA from the spleen cells was extracted, and the cDNA was subjected to PCR with specific primers for mouse T-bet (up: GGAGCGGACCAACAGCATC, down: CCACGGTGAAGGACAGGAAT), and Gata-3 (up: TCTGGAGGAGGAACGCTAATGG, down: GAACTCTTCGCACACTTGGAGACTC). The ratios for T-bet/β-actin and Gata-3/β-actin mRNA were also calculated for each sample. Meanwhile, the expression of T-bet and Gata-3 from the spleen cells were detected using Western blot.

### Splenocyte proliferation and IFN-γ^+^ T cell measurement

The spleen cells isolated from the mice were cultured and incubated with the Esat-6/3e peptides or medium alone [50]. The proliferation response of splenocytes were determined by 3-(4, 5-dimethylthiazol-2-yl)-2, 5-diphenyltetrazolium bromide (MTT) [51]. Besides, ELISPOT experiment was performed with the assay kit (DAKEWEI, China). And the splenocytes (5×10^5^ cells/well) were plated and treated as treated as above mentioned. Thereafter, the biotinylated anti-IFN-γ mAb was added for 2 h, and the plate was supplemented with streptavidin-alkaline phosphates, and the color was shown by AP-colorimetric substrate.

RETRACTED

### CTL assay in vivo

CTL assay *in vivo* was performed as described procedure [52]. Briefly, CTL target cells were prepared from the spleen of naïve mice and pulsed with the mixture of the Esat-6/3e peptides (10 µg/ml) or no peptides overnight at 4°C. Peptides-pulsed splenocytes were then labeled with a high concentration of CFSE (5 µM) or unpulsed splenocytes with a low concentration of CFSE (0.5 µM). 2.5×10^6^ pulsed and 2.5×10^6^ unpulsed splenocytes (1∶1 ratio) were mixed and transferred to the immunized mice. The splenocytes of mice at 18 h after treatments were isolated for acquisition on a FACS caliber instrument (BD Biosciences, USA). Finally, the ratio of CFSE_high_/CFSE_low_ in the vaccinated mice was compared.

### *M.tb* H37Rv challenge

Fore weeks after *M.tb* H37Rv challenge, the left lungs and spleen of mice were homogenized. Then, 100 µl of diluted samples (10^−3^, 10^−4^, and 10^−5^) were plated on agar plates and incubated for 8 weeks. The number of CFU was then counted, and the data were expressed as mean of log_10_ CFU value ± standard deviation for each group.

Besides, the lung samples of mice were subjected to hematoxylin-eosin (HE) staining for histological analysis. To score lung inflammation and damage, the sections of entire lung were observed under light microscope (LM) with software Image plus 6.0. And meanwhile, the immunohistochemistry (IHC) of the lung sections were performed with anti-CD3 or anti-F4/80 antibody staining, and the influx of T cells and macrophages (anti-CD3 and anti-F4/80 positive cells) was determined.

### Statistical analysis

Data were presented by mean ± standard deviation (mean ± SD), and analyzed using one-way ANOVA as well as multiple comparisons between groups by student's t test adjusted by Bonferroni method. A probability of *P*≤0.05 was considered statistically significant. All analysis were conducted under SAS 9.2 (SAS Institute Inc., Cary, NC, USA).

## Supporting Information

Figure S1 **The particle size distributions and zeta potential of nano-chitosan or nano-Esat-6/3e-FL plasmids were displayed.** **A.** The size and ploy dispersity of nano-chitosan and nano-Esat-6/3e-FL plasmids. **B.** The zeta potential of nano-chitosan and nano-Esat-6/3e-FL plasmids respectively.
(TIF)

Figure S2 **The nano-Esat-6/3e-FL showed high stability against DNase I.** **A.** The image showed different degradation reaction of nano-Esat-6/3e-FL and Esat-6/3e-FL with DNase I (U) digestion (1: nano-Esat-6/3e-FL+0.1U. 2: Esat-6/3e-FL+0.1U. 3: nano-Esat-6/3e-FL+0.04U. 4: Esat-6/3e-FL+0.04U. 5: nano-Esat-6/3e-FL+0.02U. 6: Esat-6/3e-FL+0.02U. 7: nano-Esat-6/3e-FL. 8: Esat-6/3e-FL). **B.** The image displayed that ratios of different volume mixture in nano-chitosan and Esat-6/3e-FL was digested by same dose of DNase I (0.1U). The lane 1 and 6 were Esat-6/3e-FL, and lane 2, 3, 4 and 5 were nano-Esat-6/3e-FL plasmids in different volume ratio of nano-chitosan and Esat-6/3e-FL (namely 1∶1, 1∶2, 1∶3 and 1∶4, respectively).
(TIF)

Figure S3 **The detection of cytopathic effect (CPE) on rat GMCs at 48 h and 72 h after transfection of nano-pGCsi-GFP and liposome-pGCsi-GFP.** **A** and **D** showed the GMCs condition after transfection of liposome-2000-pGCsi-GFP. **B** and **E** displayed the GMCs condition transfected with nano-pGCsi-GFP. **C** and **F** showed the GMCs condition after pGCsi-GFP transfection alone (magnification: 200×).
(TIF)

Figure S4 **Cell infiltration of lung sections from the mice challenged with** ***M.tb*** **was observed.** The lung sections were stained by immunohistochemistry (IHC) with anti-CD3 (**A**) or anti-F4/80 (**B**) antibody (magnification: 200×). The percentage of lung inflammation account for the entire lung sections of these mice was scored by morphometric analysis (**C**). All experiments were conducted three times, with the representative photos. The data are shown as mean ± SD (n = 6). *P<0.05, **P<0.01, ***P<0.001 versus the mice immunized with nano-chitosan or nano-pIRES or nano-FL plasmid, and the other obvious differences of the mice with different treatments were directly displayed on the figures.
(TIF)
